# Optimization of AES-128 Encryption Algorithm for Security Layer in ZigBee Networking of Internet of Things

This article has been retracted.

**DOI:** 10.1155/2022/8424100

**Published:** 2022-04-19

**Authors:** Zhonghua Luo, Keyong Shen, Rongqun Hu, Yuhan Yang, Rongchun Deng

**Affiliations:** ^1^School of Electronics and Information, Nanchang Institute of Technology, Nanchang 330044, Jiangxi, China; ^2^College of Computer Information and Engineering, Nanchang Institute of Technology, Nanchang 330044, Jiangxi, China

## Abstract

With the rapid development of network and communication technology, the interaction of various information data is more and more frequent, and people pay more and more attention to information security. The information encryption algorithm is a research hotspot in the field of information security. The Advanced Encryption Standard (AES) algorithm has been widely used in the field of information security with its high security and encryption efficiency. This paper mainly introduces the optimization of the AES-128 encryption algorithm of the security layer in ZigBee networking of the Internet of Things. By analyzing the principles of ZigBee networking and the AES encryption algorithm, the changes are optimized. In this paper, the new S-box cryptographic properties are used after analysis and calculation. The affine transformation period, the number of iteration cycles, and the algebraic expression of the S-box are improved. Its cryptographic properties are better than the S-box of the original algorithm, and the security of the algorithm is improved. In the theory of column hybrid algorithm, the computational complexity is reduced by changing the fixed polynomial, and the efficiency of the column hybrid algorithm is improved. In this paper, the performance of the improved AES algorithm is tested. The results show that, in the power consumption curve experiment, the recovery success rate of the original algorithm is about 42%, and the recovery success rate of the improved algorithm is nearly 60%. The improved algorithm is faster than the original algorithm in achieving a recovery success rate of 100%. Experimental results show that the design can accurately complete the encryption and decryption of the AES algorithm, and the performance is better than the original algorithm, which proves the overall superiority of the algorithm.

## 1. Introduction

With the in-depth development of the Internet of Things and computer technology, the “Internet of Things” era has come; information technology has always affected our work and life. While enjoying the conveniences brought by information technology, due to the openness of the Internet information system, the problem of information security is also getting more and more attention and is urgent to be solved. In many cases, the traditional security protection based on software level still can not provide enough security for the system. Hackers can attack the operating system and steal sensitive information. More and more application scenarios need to use IoT security technology to build IoT security hardware frameworks, such as industrial control security, smart car safety, and smart home security. Encryption and decryption technology plays an important role in protecting our property security, personal information, and so on. The implementation of encryption and decryption technology depends on algorithms and security mechanisms. Secure and efficient encryption and decryption algorithms and their correct application can effectively guarantee the security of the system [1].

AES algorithm has the advantages of small memory, easy to implement, ability to resist a variety of cryptanalysis attacks, and high encryption efficiency. As the next-generation data encryption standard to replace DES, the security performance of the AES algorithm is beyond doubt, but there are still defects in the initial key fixation and keyspace determination [2, 3]. In view of the important position of AES in the field of information encryption, how to improve AES algorithm has always been the focus of modern cryptography research and analysis [4]. Since the publication of the AES algorithm, it has been highly concerned by the cryptography circles at home and abroad. With the wide application of AES in various fields, the research work on all aspects of AES is also ongoing, mainly focusing on the research of algorithm security and the discussion of implementation methods. Kalaiselvi and Mangalam mainly aim at the low power consumption and high throughput of the key expansion algorithm in the AES algorithm and use the proposed high-performance architecture to minimize the power consumption and critical path delay, instead of the existing key expansion scheme of the AES algorithm; however, the design of this method is not very suitable for the Internet of Things, and the process is relatively complicated. [5]. Zhang and Parhi proposed an AES algorithm for finding all isomorphic mappings. In view of the complexity of subfield operation and isomorphic mapping in the AES algorithm, a compound field structure was selected to optimize the AES algorithm to minimize the critical path of the algorithm, but the performance of the algorithm was not superior [6]. Soltani and Sharifian implement the design of the AES algorithm through ASIC, which can reduce the hardware area occupied by the algorithm and reduce the power consumption. Although the advantages are obvious, its disadvantages can not be ignored. The design cycle of ASIC is long and the flexibility of adjusting algorithm parameters is poor [7]. With the development of society and the progress of science and technology, the development of the Internet of Things technology is changing with each passing day, and the development of the Internet of Things has made the monitoring system widely popularized. On the basis of this technology, Abane et al. designed a monitoring system based on Exynos4412 and ZigBee wireless sensor network, to complete the control and management of system temperature and humidity and hardware facilities and to improve the AES (Advanced Encryption Standard) encryption algorithm applied to the database to realize the safe storage of data [8].

This paper mainly studies the encryption of the security layer in the ZigBee network of the Internet of Things and studies the principle of the AES algorithm and secure storage by constructing an S-box with multiple anti-interference capabilities and improving the expansion efficiency of the p-extension layer, so as to realize the optimization of the AES encryption algorithm in the ZigBee network security layer. The network is optimized. The optimized AES algorithm further improves the implementation efficiency of the algorithm, adapts to the running environment with higher and higher security performance requirements, and ensures the data security of ZigBee networking in the Internet of Things. It is of great practical significance to the increasingly serious network information security problems.

## 2. Theoretical Basis and Algorithm Optimization of ZigBee Networking and AES Algorithm

### 2.1. Theoretical Basis of ZigBee Networking

#### 2.1.1. ZigBee Protocol Architecture

ZigBee networking technology is a wireless communication technology applied in short distances and at low speed; the ZigBee protocol stack is an important concept in ZigBee networking technology. It represents the interface between users and protocols. Developers who study wireless communication need to design software in the protocol stack to realize various functions of ZigBee technology. The ZigBee protocol stack is divided into two parts. IEEE 802.15.4 defines the relevant technical specifications of phy (physical layer) and MAC (medium access layer); the ZigBee protocol stack is divided into two parts, IEEE 802.15.4 defines the relevant technical specifications of phy (physical layer) and MAC (media access layer), NWK (network layer), APS (application support sublayer), etc. The ZigBee protocol stack is based on OSI (open system interconnection) seven-layer standard modes.

ZigBee physical layer is the lowest layer in OSI seven-layer standard models, and it is the foundation of the whole system. It is responsible for sending and receiving data and establishing transmission media for the communication process between devices. Its basic function can be regarded as the medium for data transmission [9]. The physical layer of ZigBee uses the unlicensed industrial scientific medicine (ISM) band, so it defines three frequency bands, including 868 MHz, 915 MHz, and 2.4 GHz. The use of these frequency bands is open source and does not need to pay any patent fees [10]. ZigBee Network Topology is as follows.

In all ZigBee, each node has two addresses: a 16-bit network address, namely, a short address, and a 64-bit media access layer address, which is a long address. When ZigBee is set up, the coordinator allocates a short address. Different short addresses represent the differences in the location of sending and receiving messages of its terminal nodes. The 64-bit long address is the factory address of each ZigBee module, which is unique and cannot be changed [11, 12].

ZigBee has two addressing modes in the communication process. The first is unicast, which generally exists between two ZigBee. For example, serial port transparent transmission is realized by unicast; the second is broadcast, in which the coordinator node sends data to routes and terminals in the network, and the header frame of the coordinator should be 0xFFFF, so as to communicate with all terminal nodes and routing equipment in the network [10] As shown in Figure 1, ZigBee has a variety of typical network topologies. Different topologies have different characteristics. They are star topology, tree topology, and mesh topology.

There is only one coordinator node in all topologies. The full-function node is the intermediate route, and the semifunctional node is the terminal. Star structure has no router, its center is a coordinator, the process of data receiving and sending is completed between the coordinator and terminal node, and two terminals need to use the coordinator as a bridge to transfer data information. The tree network structure adds router nodes on the basis of star structure so that the communication between terminals can not only be forwarded through the coordinator but also can be forwarded by the router as a medium. This network structure is malleable and can adapt to the communication needs of more functions.

Join the network through the coordinator: after the coordinator network initialization, the node can connect with the coordinator. The steps can be divided into finding the network coordinator, sending the association request command, waiting for the coordinator to process, and sending the data request command and reply.

Join the network through the existing nodes: the nodes joining the network can not only directly connect with the coordinator but also connect to the routing equipment in the network to join the network. For a node, some of them have joined the network but lost contact with their parent node (called an isolated node), and some nodes are new nodes. When it is an isolated node, the information of the original parent node is stored in its adjacent table, so it can directly send the request information to the original parent node and join the network. If the parent node has the ability to allow it to join the network, it can directly tell it the previously assigned network address, and then, it can successfully enter the network [13]; if the number of child nodes in the network where the original parent node is located has reached the maximum value, that is, the network address has been fully allocated, the parent node cannot approve its joining and can only search and join the network again as a new node [14, 15].

### 2.2. Principle of AES Algorithm

Substitution and substitution are the operation principles of encryption and decryption algorithms. Replacing the original elements with another unrelated element is called substitution. Replacement is to rearrange and combine the elements in the original text. AES encryption and decryption algorithm makes full use of substitution and substitution methods, mainly including key expansion and round transformation, so as to realize the encryption optimization of the algorithm [13]. Round transformation is the key part of encryption and decryption algorithm, which can be summarized as a linear layer, nonlinear layer, and round key encryption layer. The linear layer includes row displacement transformation and column mixed transformation, and the nonlinear layer is byte replacement. The number of round transformations is 10 [16]. Except for the last one, the other nine times include byte replacement, row displacement transformation, column mixed transformation, and round key encryption transform [17]. Next, the four main steps of round transformation and key expansion are introduced in detail.

#### 2.2.1. Byte Replacement

Byte replacement is the first step and the only nonlinear transformation in the AES encryption algorithm. Byte replacement is a transformation that needs fine processing, and its key lies in the design of the S-box. S-box is a 16 × 16 matrix, which can provide 256 kinds of transformations. In the design of S-box, the first row of the initial S-box is {00}, {01},…, {0F}, the second line is {10}, {11},…, {1F}, then the value of each byte is replaced by its inverse multiplication, and then affine transformation is performed on each element. The definition of affine transformation is shown in

(1) $$\begin{array}{c} \left[\begin{array}{c} b_{7}\\ b_{6}\\ b_{5}\\ b_{4}\\ b_{3}\\ b_{2}\\ b_{1}\\ b_{0} \end{array}\right]=\left[\begin{array}{cccccccc} 1 & 1 & 1 & 1 & 1 & 0 & 0 & 0\\ 0 & 1 & 1 & 1 & 1 & 1 & 0 & 0\\ 0 & 0 & 1 & 1 & 1 & 1 & 1 & 0\\ 0 & 0 & 0 & 1 & 1 & 1 & 1 & 1\\ 1 & 0 & 0 & 0 & 1 & 1 & 1 & 1\\ 1 & 1 & 0 & 0 & 0 & 1 & 1 & 1\\ 1 & 1 & 1 & 0 & 0 & 0 & 1 & 1\\ 1 & 1 & 1 & 1 & 0 & 0 & 0 & 1 \end{array}\right]\left[\begin{array}{c} a_{7}\\ a_{6}\\ a_{5}\\ a_{4}\\ a_{3}\\ a_{2}\\ a_{1}\\ a_{0} \end{array}\right]⊕\left[\begin{array}{c} 0\\ 1\\ 1\\ 0\\ 0\\ 0\\ 1\\ 1 \end{array}\right]. \end{array}$$

Byte replacement is to replace the byte in the state with another byte according to the S-box. The row value is determined by the high bit, and the column value is determined by the low bit. Then, according to the row and column value, the S-box is searched, and the new byte is output as the byte in the state. Each state byte is operated in turn to realize the nonlinear transformation of the byte [15, 16]. Byte substitution is expressed as

(2) $$\begin{array}{c} b_{i,j}=S\left[a_{i,j}\right]. \end{array}$$

The inverse operation of byte replacement in the decryption algorithm is called invsubbytes. The inverse operation acts on the inverse S-box; that is, the inverse transformation of the affine function is carried out first and then the multiplication inverse on the finite field.

#### 2.2.2. Row Displacement Transformation

Row displacement transformation is a linear transformation in wheel transformation, which shifts the byte in the state according to certain rules. Specifically, it keeps the first line abcd in state unchanged and the second line efgh shift left one bit to fghe, the third line ijkl to left two bits to klij, and the fourth line mnop to shift left three bits to pmno, realizing a custom linear transformation [18]. The matrix of row displacement transformation is shown in equation (3), where *N*_*b*_ is taken as 4.

(3) $$\begin{array}{c} \left[\begin{array}{c} c_{0,j}\\ c_{1,j}\\ c_{2,j}\\ c_{3,j} \end{array}\right]=\left[\begin{array}{c} b_{0,j}\\ b_{1,\left(j+1\right)\text{mod}N_{b}}\\ b_{2,\left(j+2\right)\text{mod}N_{b}}\\ b_{3,\left(j+3\right)\text{mod}N_{b}} \end{array}\right]. \end{array}$$

In the decryption algorithm, invshiftrows shifts the first row of abcd right three bits to bcda, the second line efgh to two bits to ghef, the third line ijkl to right one bit to lijk, and the fourth line mnop to remain unchanged.

#### 2.2.3. Column Mixed Transformation

The column mixed transformation is to operate on each column in the state. In the column mixed transformation, each column is regarded as a polynomial in the finite field, which is multiplied by another polynomial (*a*)*x* under module *x*^4^ + 1. The coefficients of the polynomial are selected as 01, 02, and 03. The expression of (*a*)*x* is as follows:

(4) $$\begin{array}{c} a\left(x\right)=03x^{3}+01x^{2}+01x+02. \end{array}$$

In the above formula, *a*(*x*) is the desired polynomial result. And in the concrete calculation, the column mixed transformation can be regarded as multiplying each column of the original matrix with the fixed matrix to obtain a new matrix:

(5) $$\begin{array}{c} d\left(x\right)=c\left(x\right)\left(a\left(x\right)\text{mod}\left(x^{4}+1\right)\right). \end{array}$$

The inverse transformation of column mixed transformation is inverse column mixed transformation. Similar to MixColumns, invmixcolumns also multiplies each column in the matrix with a fixed matrix:

(6) $$\begin{array}{c} \left[\begin{array}{c} d_{0,j}\\ d_{1,j}\\ d_{2,j}\\ d_{3,j} \end{array}\right]=\left[\begin{array}{cccc} 0E & 0B & 0\;D & 09\\ 09 & 0E & 0B & 0\;D\\ 0\;D & 09 & 0E & 0B\\ 0B & 0\;D & 09 & 0E \end{array}\right]\left[\begin{array}{c} c_{0,j}\\ c_{1,j}\\ c_{2,j}\\ c_{3,j} \end{array}\right]. \end{array}$$

#### 2.2.4. Round Secret Key Addition

In the round transformation, each round will generate a new round key obtained by key expansion. The XOR operation between the new round key and the state matrix is called round key addition [19]. The expression of round key addition is as follows:

(7) $$\begin{array}{c} \left[\begin{array}{c} e_{0,j}\\ e_{1,j}\\ e_{2,j}\\ e_{3,j} \end{array}\right]=\left[\begin{array}{c} d_{0,j}\\ d_{1,j}\\ d_{2,j}\\ d_{3,j} \end{array}\right]⊕\left[\begin{array}{c} k_{0,j}\\ k_{1,j}\\ k_{2,j}\\ k_{3,j} \end{array}\right]. \end{array}$$

#### 2.2.5. Key Extension

In the process of round transformation, in order to improve the computational complexity, each round needs a round key. The round key is obtained by key expansion based on the initial key. The key expansion is an irreversible nonlinear transformation. The original initial key is marked as *w*[0,3]. After the key expansion, new 40 words are generated and grouped as *w*[*i*](*I* = 4,…, 43). According to the different values of *I*, different keys are obtained. When *i* ≠ *a* multiple of 4, *w*(*i*) = *w*(*i* − 4) ⊕ *T* [*w*(*i* − 1)], T-transform is a transformation function, which includes three steps. First, the 4 bytes of each word are shifted to the left one bit in turn to confuse the original key operation. Then, the S-box is used to replace each byte in the state to reduce the correlation between the key rounds and increase the difficulty of deducing the unknown key from the known round key. Finally, the 4 bytes obtained are different from the round constant or the round constant can effectively eliminate the symmetry of cryptographic performance [20, 21].

### 2.3. Optimization of AES Algorithm

#### 2.3.1. S-Box Optimization

In this paper, we use the following S-box creation method. The S-box nonlinear transformation is *y* = (*ux*)^−1^ + *v*, and the inverse S-box nonlinear transformation is *y* = *u*^−1^(*x* + *v*)^−1^. We choose (*u*, *v*) = ({34},{*ba*}) as affine transformation pairs. Compared with the original method of creating an S-box, this improved method uses less hardware resources, faster processing speed, and better security.

On the finite field *G*(2^8^), multiplication inversion is a very complex function. If the S-box is formed in the finite field *G*(2^8^), the combinatorial logic will be very complex and the number of logic gates in the circuit will be greatly increased [22]. Therefore, according to the properties of the finite field, this paper transforms the isomorphic transformation of the finite field *G*(2^8^) and the finite field *G*[(2^4^)^2^], converts the operation of multiplication inversion in *G*(2^8^) to *G*[(2^4^)^2^], and then generates S-box, which can greatly reduce the complexity of the logical operation and the use of resources. The specific process of multiplication inversion is described as follows [23].

Firstly, the input *X* of *G*(2^8^) is mapped to the elements *b* and *c* in *G*(2^4^) by using the linear transformation *L*. Then, the first-order polynomial of the corresponding finite field *G*(2^4^) is constructed. The inverse elements *p* and *q* of the elements *b* and *c* in the finite field *G*(2^4^) can be calculated through the multiplication and inverse calculation of multiplication on the finite field *G*(2^4^). Finally, the linear transformation *L*^−1^ is constructed to map the elements *p* and *q* in the finite field *G*(2^4^) to the finite field *G*(2^8^). Thus, the inverse element *y* = *L*^−1^ (*p*, *q*) of the element *x* in the finite field *G*(2^8^) can be obtained.

According to the knowledge of finite fields, we can know that all elements in the compound field *G*[(2^4^)^2^] can express the coefficients in *G*(2^4^) by *bx* + *c* [24]. If we define the irreducible polynomial *x*^2^ + *Ax* + *B* of multiplication in the finite field *G*[(2^4^)^2^], we can verify that the inverse multiplication element of any element *bx* + *c* in *G*[(2^4^)^2^] is

(8) $$\begin{array}{c} {\left(bx+c\right)}^{-1}=b{\left(b^{2}B+bcA+c^{2}\right)}^{-1}x+\left(c+bA\right){\left(b^{2}B+bcA+c^{2}\right)}^{-1}. \end{array}$$

In formula (8), (*b*^2^*B* + *bcA* + *c*^2^)^−1^ is the inverse element of multiplication of *b*^2^*B* + *bcA* + *c*^2^ on *G*(2^8^). The logic implementation process is as follows:

(1) For the mapping from the finite field *G*(2^8^) to the compound field *G*[(2^4^)^2^], the linear change *L* is constructed according to the reduced polynomial *p*(*x*) = *x*^2^ + *Ax* + *B* in *G*(2^8^). According to formula (1), the input *x* of *G*(2^8^) is mapped to the elements *b* and *c* on *G*(2^4^), where *B* is the constant element in *G*(2^4^) and *L* is a matrix of 8 × 8. The matrix consists of 1 and 0. Matrix *L* is determined by the value of *B*, a is 1, and *B* is 8.
(2) The inverse mapping from the compound field *G*[(2^4^)^2^] to the finite field *G*(2^8^) needs to construct the linear transformation *L*^−1^; the inverse elements *p* and *q* in *G*(2^4^) map the inverse elements *Y* in *G*(2^8^), as shown in equation (9), where the multiplication of linear transformation *L*^−1^ and linear transformation *L* is *e* matrix*LL*^−1^ = *E*.
  (9) $$\begin{array}{c} Y=L^{-1}\left\{p\left[3:0\right],q\left[3:0\right]\right\}. \end{array}$$
(3) The inverse *p* and *q* of *b* and *c* are obtained by calculation in the field *G*(2^4^). Firstly, we need to construct *G*(2^4^), *q*(*x*) = *x*4 + *x* + 1 as the original polynomial of *G*(2^4^) lie and *a* (*x*), *d*(*x*), *e* (*x*) ∈ *G*(2^4^). The addition in *G*(2^4^) is based on the addition of the bit module. Multiplication is the multiplication of polynomials; then, the modulus is taken by *q*(*x*) and then calculated according to *a*(*x*) ⊗ *d*(*x*)modq(*x*). The inverse element *a*^−1^ of *a* in *G*(2^4^) is calculated by *a* × *a*^−1^ = 1modq(*x*).

The polynomial *bx* + *c* in *G*(2^4^) is constructed, and the multiplication, inversion, and addition in *G*(2^4^) are used for calculation. Finally, the inverse elements *p* and *q* of *b* and *c* in *G*(2^4^) are obtained. The following formula can be deduced:

(10) $$\begin{array}{c} {\left(bx+c\right)}^{-1}=b{\left(8b^{2}+bc+c^{2}\right)}^{-1}x+\left(c+b\right){\left(8b^{2}+bc+c^{2}\right)}^{-1},\\ p=b{\left(8b^{2}+bc+c^{2}\right)}^{-1},\\ q=\left(c+b\right){\left(8b^{2}+bc+c^{2}\right)}^{-1}. \end{array}$$

#### 2.3.2. Column Obfuscation Optimization

From the diversity of the algorithm, there are three different column confusion coefficient matrices; in the use of the algorithm, we will randomly choose one of the three to defend. There is a coefficient matrix whose inverse is itself. Let *c*(*x*) = *c*_3_*x*^3^ + *c*_2_*x*^2^ + *c*_1_*x* + *c*_0_, and a sufficient condition for *c*(*x*)*c*^−1^(*x*) = {01} is *c*_1_ = *c*_3_ and *c*_0_ + *c*_2_ = {01} so that encryption and decryption can be carried out simultaneously with only one coefficient matrix. Some scholars have shown that the chip area and processing speed of column obfuscation transform module mainly depend on matrix elements, Hamming weight, and nonzero coefficient value [25, 26]. The Hamming weight is less than or equal to 3, the number of branches is 5, and the matrix is reflexive. Considering the processing speed of coefficient matrix hardware implementation, the final optimization scheme is as follows:

(11) $$\begin{array}{c} c\left(x\right)=\left\{01\right\}x^{3}+\left\{02\right\}x^{3}+\left\{01\right\}x+\left\{03\right\}. \end{array}$$

The above is the whole process of AES algorithm optimization. Next, this paper will combine this process to carry out optimization experiments of the AES-128 encryption algorithm of the IoT security layer.

## 3. Experimental Steps and Platform of AES Algorithm Optimization

### 3.1. Optimization Experiment of AES Algorithm

The experiment is implemented on an Intel Core i5-10400 CPU and 8.0 GB memory ordinary PC platform. The key recovery algorithm is written in Verilog. AES key is generated randomly. 13 round key bytes are calculated by the key expansion formula, and the mask value of 13 bytes is randomly generated which is different from each round key byte. 185 Hamming weights of the masked bytes are used as the input of the key recovery algorithm. In this paper, we simulate the situation of obtaining multiple power consumption curves, that is, different power consumption curves generated by using the same key encryption for different plaintexts, and then, the attacker analyzes the power consumption curves to obtain the Hamming heavy information of the intermediate value. Based on the premise of a simple power consumption attack, this project does not simulate the process of device attack and directly uses the simulated mask key Hamming heavy as the attack data after a simple power consumption attack to recover the key [27] *AES Algorithm Optimization Experimental Simulation Platform*.

The simulation software used in this design is Modelsim 10.4. The software can simulate the engineering described by VHDL, Verilog, and these two hardware input languages [28]. In addition, the software can run a variety of common IEEE hardware description language standards [29]. The simulation process of Modelsim is shown in Figure 2.

1. First of all, you need to create a project and enter the name of the project and the address of the project.
2. Add the project to the project just created, and click Add existing file. Because Verilog is selected as the design language for this design, the code. V files written in advance and testbench are added to the project.
3. In the project tab, you can see the file just loaded, and then click complie in the selection menu to compile.
4. Open the work library on the library tab, right-click simulate to testenclosure file, and then add the interface needed for simulation, and then set the simulation time and click Run to run the simulation.
5. Get the simulation results, according to the simulation waveform of each interface, compare them with the expected results, and then improve the debugging.

## 4. Performance Test and Comparison of AES Encryption Algorithm after Optimization

### 4.1. AES Encryption and Decryption Speed Test

Through the above theoretical analysis, firstly, the AES encryption algorithm is implemented, and its encryption speed is tested. The test content includes documents, pictures, images, and other different data. As shown in Table 1, the AES encryption and decryption speed test table is listed.

As shown in Figure 3, the time spent by the AES encryption algorithm in data encryption and decryption is gradually increased according to the increase of data volume in turn. Moreover, the encryption time of the AES symmetric encryption algorithm is similar to encryption, which is because the decryption process of the AES algorithm is the reverse operation of the encryption process, and its algorithm has no change. In the process of encryption and decryption, the most time-consuming is the loading speed of data, which is much higher than that of the AES encryption algorithm. Because of the limitation of PC function, it will take more time to read relatively large files [30].

At the same time, AES symmetric encryption algorithm takes a long time to encrypt and decrypt, which has nothing to do with the content of the encrypted data. The encryption and decryption time of documents, pictures, video, and other data is similar in the same size.

### 4.2. Experimental Results and Comparison of AES Optimization Algorithm Power Consumption

As shown in Table 2, it is the experimental results of the improved algorithm. Each row represents the key recovery results under different power consumption curves. The amount of information obtained by different power consumption curves is different, so the recovery results are also different. Because the time-consuming of the recovery experiment can not be predicted, the timeout time is set. According to the different attack conditions, the timeout period from 90 s to 450 s is set. If the time exceeds, the experiment will be stopped as shown in Table 2.

Table 2 shows the experimental results of the algorithm. For example, the first line represents the experimental results of obtaining five power consumption curves. Setting the timeout time to 450 s, a total of 23 experiments have been carried out. The recovery success rate is 58.9%, the average time consumption is 78.6 s, and the average residual entropy is 7.8 bit. The rest of the experimental data are the same.

#### 4.2.1. Comparison of Recovery Success Rate

As shown in Figure 4, under the condition of 5 power consumption curves, the recovery success rate of the original algorithm is about 42%, and the recovery success rate of the improved algorithm proposed in this paper is nearly 60%; in the case of 15 power consumption curves, the recovery success rate of the improved algorithm reaches 100%, while that of the original algorithm reaches 100% under the condition of 30 power consumption curves. In the recovery success rate, the improved algorithm is better than the original algorithm.

#### 4.2.2. Comparison of Average Time Consumption

As shown in Figure 5, in the case of 5 power consumption curves, the average time consumption of the improved algorithm is 78.6 s, and the average time consumption of the original algorithm is as high as 370 s; while in the case of 10 power consumption curves, the average time consumption of both the improved algorithm and the original algorithm is greatly reduced. The more the power consumption curve is, the smaller the average time consumption of the algorithm is, which accords with the analysis before the experiment [31–33].

#### 4.2.3. Average Residual Entropy

As shown in Figure 6, it is the comparison of the average residual entropy of the algorithm. In five power consumption curves, the average residual entropy of the original algorithm is higher than that of our proposed algorithm, while the average residual entropy of the proposed algorithm is slightly higher than that of the original algorithm.

### 4.3. Experimental Comparison Based on Data Decomposition

#### 4.3.1. Encryption Performance of Input Plaintext Data before and after Decomposition

As shown in Table 3 and Figure 7, compared with the original algorithm encryption program, the running time of the improved algorithm encryption program is significantly shortened, and the performance is greatly improved. Moreover, with the increase in data volume, the performance improvement is more obvious.

#### 4.3.2. Decryption Performance of Input Plaintext Data before and after Decomposition

As shown in Table 4 and Figure 8, under the condition of input plaintext data decomposition, the performance of the encryption program and decryption program is roughly similar. The running time of the improved algorithm is shorter than that of the original algorithm, and the larger the amount of data, the greater the performance gap.

This experiment is over now. According to the above experimental content, the experimental conclusion drawn in this paper is as follows: after the improvement of the AES optimization algorithm, the running time of the encryption program of the AES-128 encryption algorithm of the Internet of Things security layer is significantly shortened, and the performance of the algorithm is significantly shortened. It has also been greatly improved, and the more the input data, the more obvious the performance improvement of the algorithm.

## 5. Conclusions

The information encryption algorithm is an important means to prevent information leakage in the transmission process and ensure information security. In this paper, according to the AES algorithm of security layer in ZigBee network of the Internet of Things, through the investigation and analysis of various optimization implementation methods of AES, this paper puts forward an implementation method of AES algorithm which can be used for resource reuse in ZigBee networking. The improved AES algorithm proposed in this paper has the characteristics of low cost, small consumption, good stability, and high security. Compared with the original algorithm and other algorithms, it has achieved good results.

This paper discusses the technical details of ZigBee networking, analyzes the theoretical basis of the AES encryption algorithm in detail, and optimizes the AES encryption algorithm according to the technical characteristics of ZigBee networking. From the perspective of algorithm optimization, this paper optimizes the S-box in the original AES algorithm and improves the cryptographic properties of the S-box by selecting the optimal affine transformation pairs, thus, improving the security of the algorithm; the optimization of MixColumns is to select *c*(*x*) = {01}*x*^3^ + {02}*x*^3^ + {01}*x* + {03} as fixed polynomial of column confusion so that encryption and decryption can be realized with the same matrix. This paper uses the improved algorithm and the original algorithm for performance comparison experiments; after the overall analysis and verification of the results, it shows that the design has good performance in data encryption processing.

In this paper, the improved AES algorithm has some advantages compared with the original algorithm, but there are still some shortcomings in the current work. For example, there is room for innovation in research methods and content. In the future, we will study and improve the implementation of the AES algorithm in the following aspects: we further improve the processing speed of encryption and decryption of the AES algorithm; we implement a lightweight AES algorithm for the security architecture of the Internet of Things through the cooperation of software and hardware.

## Figures and Tables

**Figure 1:** Three network topologies.

**Figure 2:** Modelsim simulation process.

**Figure 3:** AES encryption and decryption speed test chart.

**Figure 4:** Comparison of the recovery success rate of three algorithms.

**Figure 5:** Comparison of three average time-consuming algorithms.

**Figure 6:** Comparison of average residual entropy of three algorithms.

**Figure 7:** Comparison of encryption performance of input plaintext data before and after decomposition.

**Figure 8:** Comparison of decryption performance of input plaintext data before and after decomposition.

**Table 1:** AES encryption and decryption speed test.

Serial number	File size (MB)	Read time (ms)	Encryption time (ms)	Decryption time (ms)
1	0.5	129	38	86
2	1	204	43	87
3	4	386	58	127
4	10	478	126	181
5	24	937	281	374

The encryption and decryption test mainly uses 0.5 mb–24 mb data.

**Table 2:** Experimental results of improved algorithm.

Power consumption curve number	Time out (s)	Number of experiments	Recovery success rate	Average time spent (s)	Average residual entropy (bit)
5	450	23	58.9	78.6	7.8
10	240	500	84.3	26.7	4.1
15	90	500	100	1.13	1.4
20	90	500	100	0.26	0.98
30	90	500	100	0.09	0.27

**Table 3:** Encryption performance comparison table of input plaintext data before and after decomposition.

*N*	T1	T2	T3
10000	12341	7845	6723
20000	24859	15967	10285
30000	38412	20379	18436
40000	49836	27841	24189
50000	66218	36194	35102

**Table 4:** Comparison table of decryption performance of input plaintext data before and after decomposition.

*N*	T1	T2	T3
10000	13842	8034	7542
20000	26125	16230	14657
30000	38436	21894	19751
40000	55102	31642	30984
50000	69024	38976	36481

## Data Availability

No data were used to support this study.
